RETRACTED

# Modulation of Signal Proteins: A Plausible Mechanism to Explain How a Potentized Drug Secale Cor 30C Diluted beyond Avogadro's Limit Combats Skin Papilloma in Mice

**DOI:** 10.1093/ecam/nep084

**Published:** 2011-06-18

**Authors:** Anisur Rahman Khuda-Bukhsh, Soumya Sundar Bhattacharyya, Saili Paul, Suman Dutta, Naoual Boujedaini, Philippe Belon

**Affiliations:** ^1^Cytogenetics and Molecular Biology Laboratory, Department of Zoology, University of Kalyani, Kalyani 741235, West Bengal, India; ^2^Boiron Laboratory, Lyon, France

## Abstract

In homeopathy, ability of ultra-high diluted drugs at or above potency 12C (diluted beyond Avogadro's limit) in ameliorating/curing various diseases is often questioned, particularly because the mechanism of action is not precisely known. We tested the hypothesis if suitable modulations of signal proteins could be one of the possible pathways of action of a highly diluted homeopathic drug, Secale cornutum 30C (diluted 10^60^ times; Sec cor 30). It could successfully combat DMBA + croton oil-induced skin papilloma in mice as evidenced by histological, cytogenetical, immunofluorescence, ELISA and immunoblot findings. Critical analysis of several signal proteins like AhR, PCNA, Akt, Bcl-2, Bcl-xL, NF-*κ*B and IL-6 and of pro-apoptotic proteins like cytochrome *c*, Bax, Bad, Apaf, caspase-3 and -9 revealed that Sec cor 30 suitably modulated their expression levels along with amelioration of skin papilloma. FACS data also suggested an increase of cell population at S and G2 phases and decrease in sub-G1 and G1 phages in carcinogen-treated drug-unfed mice, but these were found to be near normal in the Sec cor 30-fed mice. There was reduction in genotoxic and DNA damages in bone marrow cells of Sec Cor 30-fed mice, as revealed from cytogenetic and Comet assays. Changes in histological features of skin papilloma were noted. Immunofluorescence studies of AhR and PCNA also suggested reduced expression of these proteins in Sec cor 30-fed mice, thereby showing its anti-cancer potentials against skin papilloma. Furthermore, this study also supports the hypothesis that potentized homeopathic drugs act at gene regulatory level.

## 1. Introduction

Convincing positive effects of homeopathic drugs in prevention and treatment of various cancers like prostate [1], liver [2–5] and Ehrlich ascites carcinoma and Dalton's lymphoma [6, 7] have been documented earlier in laboratory animals. However, the mechanisms of chemoprevention or intervention by homeopathic remedies have been debated over and again and some critics even suggested that the actions of these drugs are no better than the “placebo” effects [8, 9].

In recent past, clinical trials and laboratory-based experiments have provided evidences that these drugs interfere with cancerous growth through genetical and physiological pathways [10–12].

RETRACTED

However, despite scientific evidences and arguments for and against the efficacy of potentized homeopathic drugs diluted beyond Avogadro's limit (potency 12 and above), the issue has not yet been fully resolved, particularly because such ultra-high diluted drugs cannot theoretically have even a single molecule of the original drug substance. But more recent works [6, 7, 13] pointing to the ability of highly diluted (dynamized) drugs showing positive effects on the face of their physical non-existence have reopened the search for other possible molecular pathways of activities. Sunila et al. [6, 7] addressed this issue in *in vitro* experimental model (cancer cell line) and suggested that potentized homeopathic drugs diluted beyond Avogadro's limit can modulate certain signal proteins.

Analysis of expression of signal proteins, one of the state-of-the art techniques to understand signaling pathways [14], has been employed to understand the mechanism of chemoprevention or intervention by anti-cancer drugs employing HeLa cancer cell line [15, 16]. However, the exact signaling pathway through which they possibly act still remains rather obscure.

With this view in mind, the present work was aimed at testing the hypothesis if (i) Secale cornutum 30C (Sec cor-30, diluted 10^60^ times) could show amelioration of skin cancer and (ii) to examine if some relevant signal proteins were suitably modulated during this process. This drug was chosen because Sec cor-30 is claimed in homeopathic literature [17] to have great action against any stubborn case of skin lesions, particularly of hemorrhagic and wrinkled ulceration of skin. A DMBA + croton oil-induced mouse skin cancer model was chosen for this study, primarily because the cytokine-mediated cell signaling pathway is well defined in this model. DMBA is known to induce skin cancer through ligand-activation of the Aryl hydrocarbon receptor (AhR) [18–20] and by up-regulation of proliferating cell nuclear antigen (PCNA) [21, 22]. Thus, the study of expression of other downstream proteins like IL-6, NF-*κ*B, Bcl-2, Bcl-xL, Bad, Bax, p53, caspase-3 and -9 could throw significant light on the pathway of carcinogenesis by DMBA + croton oil application. Furthermore, this could highlight how the homeopathic drug could, if it did, combat the carcinogenesis process.

## 2. Methods

Inbred Swiss albino mice (*Mus musculus*) of both genders reared in the animal house under standard hygienic conditions and food were used. The experiments were performed with clearance from the Ethical Committee, University of Kalyani and as per the stipulated guidelines. Healthy mice 8–10 weeks old, weighing between 22 and 26 g were selected randomly for use in the experiment. The selected mice were allocated to four groups, each comprising six mice (in two replicates of three mice each kept in separate cages).

RETRACTED

**Group 1 (Negative control)**

mice fed with normal diet and water *ad libitum* without any exposure to DMBA + croton oil.

**Group 2 (Treated)**

100 *μ*g of DMBA was applied once a week and 1% croton oil was applied twice a week to skin on dorsal side of the mouse for 24 weeks. Instead of the generally adopted practice of treating mice with DMBA for once or twice a week for 4 weeks (for initiation) [23], followed by regular application of croton oil (for promotion of papilloma) [24] as a complete carcinogenesis protocol, the mice in the present investigation were repeatedly treated with DMBA, once every week for 24 weeks, because: (i) that would further ensure development of papilloma (with possibility of many of them turning malignant) and (ii) we were interested in conducting studies on modulation of signal protein expression (particularly AhR), if any, as a result of DMBA and croton oil treatment, and any further modulation caused by the homeopathic drug [25]. DMBA is known to activate AhR by acting as a ligand.

**Group 3 (positive control)**

100 *μ*g of DMBA was applied once a week and 1% of croton oil was applied twice a week to skin on dorsal side of the mouse for 24 weeks and fed a daily dose (two times) of Alcohol-30C, (Alc-30; placebo) through gavage with the aid of a fine tube.

**Group 4 (drug-fed)**

this group was similarly treated as in Group 2 but, in addition, they were treated with Sec cor-30. Each mouse was fed a daily dose (two times) of 0.06 ml of stock solution of Sec cor 30 through gavage with the aid of a fine tube.

### 2.1. Preparation of the Potentized Sec cor 30

The potentized homeopathic drug, Sec cor 30 was procured from HAPCO (BB Ganguly Street, Kolkata). The placebo, Alc-30, was prepared from the same stock of alcohol used for preparation of Sec cor 30, as per the standard procedure of homeopathic principle of “succussions and dilution.” One milliliter of each of Sec 30 and Alc-30 was diluted separately with 20 ml of double distilled water to make the stock solution of Sec 30 and Alc-30, respectively.

### 2.2. Incidence of Skin Tumors

The numbers of tumor formation in four groups were recorded weekly.

### 2.3. Histology and Immunofluorescence

Back skin samples were dissected from the lesion and/or tumor regions of the mid-dorsal back skin of both the drug-fed and positive controls (and also of normal back skin of negative control) and fixed in normal buffer formalin, followed by dehydration treatment, as per the standard practice [21]. After storing at room temperature for less than a week in 70% alcohol, the tissues were washed two times each for 30 min in xylene, and then transferred to the embedding bath. The paraffin blocks were cut into ribbon like pieces and placed on to slides after stretching into warm water. The paraffin was removed by xylene (two washes each for 10 min), then the xylene was removed by alcohols. Processed tissues were stained in haematoxylin for 2 min, followed by washing in distilled and tap water, respectively. Then tissues were brought into alcohol medium (70%, 90% two washes each for 2 min), followed by staining with eosin (30 s) and dehydrated into 90% and absolute alcohol (two washes each for 2 min). Finally, xylene treatment (two washes each for 2 min) was carried out, followed by mounting into DPX. For immunofluorescence study, the technique of Arabzadeh et al. [26] was adopted with a little modification. Briefly, cut tissue sections were de-paraffinized and incubated separately for 12 h with mouse monoclonal AhR and PCNA antibodies, respectively, procured from Abcam International, USA. Then after blocking with 3% BSA, the tissue sections were incubated for 2 h with fluorescence isothiocyanite (FITC) conjugated secondary antibody purchased from Sigma, St. Louis, MO, USA. The fluorescence intensity of FITC was measured under ZEISS fluorescence microscope, Germany, Carl Zeiss MicroImaging, Inc., Thornwood, New York.

RETRACTED

### 2.4. Signal Proteins

These were either detected by ELISA method (caspase-3) or by western blots (the remaining ones).

#### 2.4.1. Western Blot

It was performed as per protocol described previously [27]. Briefly, mouse skin tissues were homogenized in lysis buffer containing 50 mM Tris-HCl, pH 8.0, 1% Nonidet P-40, 125 mM NaCl, 1 mM NaF, 1 mM phenylmethylsulfonyl fluoride, 1 *μ*g ml^−1^ aprotinin, 1 mM Na_3_  VO_4_ and 10 mM sodium pyrophosphate [14]. Equal amount of protein as determined by Lowry assay [28] were diluted with 5× sample loading buffer, boiled and loaded onto 12% polyacrylamide gels. After electrophoresis, the protein bands were transferred to a nitrocellulose membrane, and membranes were blocked in 5% milk in 1 × TBS, 0.05% Tween, then the transferred bands of AhR, PCNA, p53, Bcl-2, Bcl-xL, Bad, Bax, NF-*κ*B (p65 sub-unit of nuclear extract), cytochrome *c*, IL-6 and caspase-9 were bound to their respective monoclonal antibodies purchased from Abcam, Kendall Square, Cambridge, USA and Santa Cruz Biotechnology Inc., Santa Cruz, CA, USA. Antibodies for caspase-9, Akt and cytochrome *c* were purchased from BD Bioscience, San Jose, CA USA. The bound proteins were treated with the appropriate ALP-conjugated secondary antibodies (Sigma Chemicals, St. Louis, MO, USA). The same membranes were also immunoblotted against *β*-actin (house-keeping protein) for data normalization. For quantitative analysis of each band, density was determined using Gel Doc System; Ultra Lum, East Uwchlan Ave, Exton, PA, USA; Nonlinear Dynamic Ltd, Newcastle, UK.

RETRACTED

#### 2.4.2. ELISA

The activity of caspase-3 was measured using the colorimetric substrate method from skin tissue employing an ELISA reader (Thermo Scientific, Vantaa, Finland), following Das et al. [24]. Cytosolic extracts were prepared by homogenization of dorsal shaved area of skin tissues in extraction buffer containing 25 mM HEPES (pH 7.5), 5 mM MgCl_2_, 1 mM EDTA, 0.1% (w/v) CHAPS and 10 *μ*g aprotinin. Subsequently, the homogenates were centrifuged at 13 000 × g for 15 min at 4°C. The supernatant fraction was used to determine caspase-3 activity. In brief, caspase-3 colorimetric substrates (Ac-DEVD-pNA), procured from Sigma, were incubated with cell lysates for 1 h at 37°C, then the amount of chromophore, p-nitroaniline (p-NA), released by caspase-3 activity was quantified by measuring the optical density at 405 nm. Caspase-3 activity was expressed as *μ*M p-NA released per hour per milligram cellular protein.

### 2.5. Cytogenetic Assay

The standard cytogenetic protocols like assays of chromosome aberrations (CA), micronuclei (MN), mitotic index (MI) and sperm head anomaly (SHA) have been adopted in the present study [2, 3].

#### 2.5.1. CA

Slides were prepared by the conventional flame-drying technique followed by Giemsa staining for scoring bone marrow CA. A total of 300 bone marrow cells were observed.

#### 2.5.2. Micronucleus Preparation

One part of the suspension of bone marrow cells in 1% sodium citrate was smeared on clean grease-free slides, briefly fixed in methanol and subsequently stained with May-Grunwald followed by Giemsa. Approximately 3000 bone marrow cells, comprising both polychromatic erythrocytes and normochromatic erythrocytes were scored.

#### 2.5.3. MI

It was determined from the same slide that was scanned for MN, and a total of 5000 cells were examined from each series. The non-dividing and dividing cells were recorded and their ratios ascertained.

#### 2.5.4. SHA

The technique of Wyrobek [29] was adopted. 5000 sperms were examined in each series.

#### 2.5.5. Estimation of DNA Damage

Comet assay was performed with single-cell gel electrophoresis, as per protocol described elsewhere [30]. Briefly, peripheral blood nuclear cells (PBMC) (1 × 10^4^) were suspended in 0.6% low-melting agarose and layered over a frosted microscopic slide previously coated with a layer of 0.75% normal-melting agarose to ensure firm gripping. The slides were then kept at 4°C for solidification. Subsequently, slides were immersed in a lysis buffer of pH 10 and kept overnight for lysis of cell and nuclear membranes. The following day slides were transferred into a horizontal electrophoresis chamber containing electrophoresis buffer (300 mM NaOH, 1 mM Na_2_EDTA; pH 13.0) and presoaked for 20 min in order to unwind DNA. Electrophoresis was then carried out for 20 min (300 mA, 20 V). Slides were then washed thoroughly with neutralizing buffer (Tris 0.4 M, pH 7.5), stained with ethidium bromide (final concentration of 40 *μ*g ml^−1^) and examined under a Lyca fluorescence microscope. The percentage of DNA breakage was determined by measuring the comet tail length using the software Motic Image China.

RETRACTED

#### 2.5.6. Cell-Cycle Analysis

Cellular DNA was stained with propidium iodide and quantified by flow cytometry according to Nicoletti's procedure [31]. Briefly, cells were fixed with 70% (v/v) cold aqueous ethanol (−20°C) and stored at 4°C for at least 24 h. The cells were washed in phosphate buffer saline, after cell centrifugation, cell pellets were stained with propidium iodide staining solution containing 10 *μ*g   ml^−1^ propidium iodide, 5 K units of RNase, and 0.1% (v/v) Triton X-100. The cell suspension was incubated in the dark at room temperature for 30 min. DNA content was determined by using a FACS Calibur flow cytometer (Becton Dickinson, Mountain View, CA). A total of 40 000 events were acquired, and MOD-FIT LT software (Becton Dickinson) was used.

### 2.6. Statistical Analysis

The significances of differences between data of carcinogen plus 2% alcohol administered mice and carcinogen administered Sec cor 30-fed mice were analyzed by the Student's *t*-test. For all quantitative analyses, data were expressed as mean values obtained from triplicate experiments (on blot and immunofluorescence studies) showing standard errors and levels of significance. Additionally, the data were also analyzed using one-way ANOVA (Turkey Method; SPSS version 11).

## 3. Results

### 3.1. External Morphology

The changes in external morphology of skin in mice subjected to: (i) no treatment (Figure 1(a); negative control: Group 1), (ii) carcinogen treatment (Figure 1(b); Group 2), (iii) carcinogen plus alcohol treatment (Figure 1(c); Group 3) and (iv) carcinogen plus Sec cor 30 treatment (Figure 1(d); Group 4) have been provided. While Groups 2 and 3 mice showed distinct growth of papilloma, both the Sec cor 30-fed groups showed much less growth of papilloma as well as loss of hair than their counterparts who did not receive Sec cor 30 treatment. The incidence of papilloma growth in different weeks in control and treated mice has been provided in Figure 2. Papillomas observed in DMBA + croton oil-treated group were significantly bigger in size (70% papillomas of ≥2.5 mM in diameter) as that of drug-fed series (8%–10%).

RETRACTED

### 3.2. Histology

As compared to the skin section with normal histological features (Figure 3(a)), irregular distribution of different cell types (e.g., squamous epithelial cells) and finger-like projections (papilloma) indicative of cancerous growth were found in the skin sections of DMBA administered mice (Figure 3(b)). Tumors of animal belonging to DMBA + croton oil-treated group were composed of focal proliferation of squamous cells, presence of some necrotic cells, keratinization and epithelial pearls, indicative of the malignant nature of tumors that is characterized by well-differentiated squamous cell carcinoma. On the other hand, in the Sec cor 30-fed mice, these features were visible to a much lesser extent (Figure 3(c)).

### 3.3. Immunofluorescence Studies

The AhR-specific immunochemical staining reveals lack of expression in normal skin (Figure 3(d)), while in DMBA-treated mice, AhR receptor was seen to take up higher level of green fluorescence in DMBA-treated mice without Sec cor 30 feeding (Figure 3(e)), indicating localization of AhR protein in carcinogen-treated mice, while in Sec cor 30-fed mice, the intensity of fluorescence was much less (Figure 3(f)). Immunofluorescence analysis for PCNA was also used to assess the proliferation activity in normal (Figure 3(g)), carcinogen-treated (Figure 3(h)) and in Sec cor 30-fed groups (Figure 3(i)) during tumor promotion. PCNA is a proliferating cell nuclear antigen associated with S phase of DNA replication. It was observed through immunofluorescence localization that PCNA expression was higher in DMBA administrated group, a characteristic intense staining, as compared to control, was observed (Figure 3(h)) and, also, there was a significant modulation of this expression in Sec cor 30-fed mice. The data on proportion of fluorescence intensity represented in Figure 3(h) prepared from three replicates would also validate the above observation.

### 3.4. Immunoblots

The expression of different signal proteins in normal healthy mice (Group 1) can be observed in the lane 1 of Figure 4. Of these, the expression level of *β*-actin, AhR, Akt, IL-6, NF-*κ*B, PCNA, Bcl-2 and Bcl-xL was of low level, while it was moderate in Bad, Bax, cytochrome *c*, Apaf, p53 and caspase-9. In the DMBA + croton oil-induced mice, the expression levels were increased in AhR, Akt, IL-6, NF-*κ*B, PCNA, Bcl-2 and Bcl-xL, while in the carcinogen administered Sec cor 30-fed mice (Group 4), there was suppression of the enhanced expression of these signal proteins. Correspondingly, there was decrease in expression of proteins like Bad, Bax, Apaf, cytochrome *c*, caspase-9 and p53 in the DMBA + croton oil-induced mice, which were increased in the Sec cor 30-fed mice. Quantification of proteins was done by densitometry using image analyzer, shown in Figure 5.

RETRACTED

### 3.5. Caspase-3 Activity through ELISA

The caspase-3 activity was higher in Sec cor 30-fed mice as compared to the DMBA-administered mice (Figure 6).

### 3.6. Cytogenetical Studies

The frequency distributions of CA, MN have been provided in Table 1. While the percentage of CA, MN, MI and SHA (Figure 7) were significantly elevated in the DMBA-induced mice as compared to normal untreated control, the values were significantly decreased by the feeding of Sec cor 30. The same was supported by the data of Comet assay (Figure 7) that indicated a much more amount of broken DNA in mice treated with DMBA + croton oil, but much less in the Sec cor 30-fed mice.

### 3.7. Cell-Cycle Analysis by FACS

The FACS analysis revealed that in the Sec cor 30-fed mice, the cell cycle was arrested more in the sub-G1 stage (32%) than that of the DMBA treated mice (23%). Furthermore, DMBA showed higher percentage of S phase (25%) in contrast to the Sec cor 30 that showed 19% of cells in S phase (Table 2).

## 4. Discussion

As far as authors are aware, this is the first demonstration where a potentized homeopathic drug diluted beyond Avogadro's limit, Secale cor 30, successfully reduced the incidence of DMBA-induced skin papilloma in mice. The histological features of skin of the drug-fed group showed evidence of amelioration rendered by the administration of the homeopathic drug. Similar findings of amelioration were also reported in case of other types of cancer like liver in mice through the administration of some crude plant extracts used as homeopathic mother tincture [2, 3] or in skin cancer by an anti-mitotic agent like 4-demethyl epipodophyllotoxin [32].

DMBA is a pro-carcinogen that requires metabolic conversion to its ultimate carcinogenic metabolite 3,4-dihydrodiol-1,2-epoxide [33]. These metabolites damage DNA presumably by formation of adducts, which could be evidenced by the increase in comet tail lengths and elevated frequencies of chromosomal aberrations in the carcinogen-administered mice. The DNA damage, CA and, consequently, disorder in metabolic functioning, contributed to the initiation of the tumorigenic process, through generation of ROS. The generation of ROS contributed further to the up-regulation of several downstream signaling proteins like NF-*κ*B, Akt and PCNA. Up-regulation of NF-*κ*B would induce the anti-apoptotic Bcl-2 and Bcl-xL genes through up-regulated Akt and thereby prevent the cells to undertake the apoptotic pathway via down-regulation of pro-apoptotic genes Bad, Bax and Apaf, caspase-3 and -9.

RETRACTED

The AhR is known to be involved in the induction of several enzymes that participate in xenobiotic metabolism. Induction of enzymes involved in xenobiotic metabolism occurs through binding of the ligand-bound AhR to xenobiotic response elements in the promoters of gene for these enzymes [34, 35]. The AhR protein contains several domains critical for function and act as a variety of transcription factors. Two PAS domains are also present in AhR, PAS-A and PAS-B [36]. The ligand-binding site of AhR is contained within the PAS-B domain and contains several conserved residues critical for ligand binding [37]. There is also a Q-rich domain located in the C terminal region of the protein and is involved in the co-activator recruitment and trans-activation [38].

Toxicity results from two different ways of AhR signaling. The first is a function of the adaptive response in which the induction of metabolizing enzymes result in the production of toxic metabolites, as for example the PAH, benz[a]pyrine, a hydrocarbon for AhR induces its own metabolism and bioactivation to toxic metabolites via the induction of CYP1A1 and CYP1B1 in several tissues [18]. The second approach to the toxicity is the result of aberrant changes in global gene transcription beyond those observed in the “AhR gene battery.”

Our present findings agree well to the reported fact that the DMBA-induced cell signaling mechanism is mediated by up-regulation of AhR. Our studies on several anti-oxidant markers like catalase, superoxide dismutase, lipid peroxidation and reduced glutathione (results unpublished) also suggested that there was the generation of reactive oxygen species (ROS) on application of DMBA. We found up-regulation in expression of some genes like IL-6, NF-*κ*B, Bcl-2 and Bcl-xL that may be responsible for leading to proliferation of cells, which in turn is reflected on an increase in PCNA in the drug-untreated mice. The increase in PCNA was accompanied by down-regulation of p53, Bax and caspase-3 genes, for which epidermal skin cells (keratinocytes) started uncontrolled divisions to subsequently form papilloma. The immunochemical localization also suggested that there was excess amount of the enzymes involving the products of unregulated genes.

Interestingly, in the drug-fed mice, very clear indication of modulation in the expression of the genes was noticed. The AhR expression was significantly lowered. Significant changes were also noted in the expression of IL-6, NF-*κ*B, Bcl-2, Bcl-xL and PCNA, which were reversed. Secale cor 30 administration caused up-regulation in the expression of p53, Bax, Apaf, caspase-3 and -9 and down-regulation of PCNA. This was a good indicator of the lower state of proliferation of the cells. This was further confirmed by our analysis of the FACS data, which showed more number of cells in the sub-G1 and G1 stages of the cycle. This tempted us to believe that the potentized homeopathic drug Sec cor-30 was possibly tagged in an unknown manner to some regulatory proteins. This binding with an unknown protein could give it the ability to bind on the AhR, thereby competitively reducing space for DMBA-binding that was responsible for lowering activity of AhR in the drug fed mice. Alternatively, it prevented the conversion of DMBA into the lesser amount of carcinogenic metabolites. Thus, the homeopathic drug apparently fulfilled the function of `ligand' by its ability to modulate the AhR activity. This was further confirmed by results of our immunofluorscence assay. Incidentally, nanoparticles associated with molecules of drug substance have been shown to affect the physicochemical property of potentized homeopathic drugs [15]. Nanoparticles of glass vial and other containers are also known to form complexes with various proteins and in some cases, in the process change their physicochemical properties [39]. Therefore, it is possible that the potentized homeopathic drug Secale cor 30, theoretically devoid of the presence of even a single molecule of the original drug substance, was still capable of apparently initiating binding to AhR, presumably through some activated proteins, because it is a pre-condition for Ahr to be ligand-activated before it could stimulate downstream proteins. However, the other possibility that cannot be excluded is the ability of Sec cor 30 to have regulatory influences on the other gene products directly or through indirect means. But one thing is clear from this study that potentized homeopathic drug does elicit regulatory influences on expression of certain relevant genes that can interfere with the carcinogenic effect of DMBA + croton oil in ameliorating/protecting skin cells from being transformed into skin papilloma (as evidenced from the difference in expression of several signal proteins), although one may still argue that it is difficult to attribute the biochemical differences between tumor and normal cells to a causal mechanism or secondary consequences for cell transformation. Therefore, further in-depth study, preferably with global micro-array methodology, may transpire that expression of many other relevant downstream protein genes can also be modulated. Incidentally, like what has been found in the present study in regard to specific signal proteins, modulation of some 147 downstream genes by a homeopathic drug has been reported by analysis of microarray [40], giving much credentials to the postulation of Khuda-Bukhsh [10–12, 41].

RETRACTED

## Figures and Tables

**Figure 1:** External morphology of skin of mice: (a) normal; (b) DMBA + croton oil; (c) DMBA + croton oil + alcohol; (d) DMBA + croton oil + Sec cor 30.

**Figure 2:** Number of tumors/mouse plotted as a function of weeks on test. Each value represents the mean number of tumor per mouse. **P < .01, ***P < .001.

**Figure 3:** Histology of skin stained with Haematoxylin/Eosin: (a) normal, (b) DMBA + croton oil + alcohol, (c) DMBA + croton oil + Sec cor 30-fed; immunofluorescence expression of AhR protein: (d) normal, (e) DMBA + croton oil + alcohol, (f) DMBA + croton oil + Sec cor 30-fed; and PCNA protein localization: (g) normal, (h) DMBA + croton oil + alcohol, (i) DMBA + croton oil + Sec cor 30-fed; (j and k) represent proportion of average fluorescence intensity of AhR and PCNA protein in different groups. **P < .01.

**Figure 4:** Immunoblots of *β*-actin, AhR, Akt, IL-6, NF-*κ*B, PCNA, Bcl-2, Bcl-xL, Bad, Bax, Apaf and p53, caspase-3 and cytochrome *c*. Ln1 represents normal; Ln2 represent DMBA; Ln3 represents DMBA + croton oil + alcohol; Ln4 represents DMBA + croton oil + Sec cor 30.

**Figure 5:** Densitometric data expressed as mean ± SE of the three independent experiments; *P < .05, **P < .01, ***P < .001. of *β*-actin, AhR, Akt, IL-6, NF-*κ*B, PCNA, Bcl-2, Bcl-xL, Bad, Bax, Apaf, p53, cytochrome *c* and caspase-9. Each experiment is representative of three different sets of experiments. Ln1 represents normal; Ln2 represents DMBA + croton oil; Ln3 represents DMBA + croton oil + alcohol; Ln4 represents DMBA + croton oil + Sec cor 30.

**Figure 6:** Showing ELISA assay of caspase-3. The rate of Ac-DEVD-pNA cleavage was measured at 405 nm. Value represents mean ± SE (*n* = 3); ***P < .001., represent highly significant differences from alcohol control.

**Figure 7:** Showing percentage of CA, MN, MI, SHA and DNA damage in different groups.*P <  .05, **P <  .01.

**Table 1:** Percentage of CA, MN in normal, DMBA + croton oil, DMBA + croton oil + alcohol and DMBA + croton oil + Sec cor 30-fed series.

Series	Major CA (%)	Other CA (%)	Total CA (%)	MN (%)
Normal	2.45	2.15	4.60 ± 0.40	0.225 ± 0.08
DMBA + croton oil	12.1	9.7	21.8 ± 0.54	1.13 ± 0.09
DMBA + croton oil + alcohol	14.0	10.3	24.3 ± 0.67	1.22 ± 0.05
DMBA + croton oil + Sec cor 30	10.0	6.67	16.67 ± 1.02**	0.68 ± 0.06**

MCP-1, monocyte chemoattractant protein-1; VCAM-1, vascular cell adhesion molecule-1; TGF-*β*_1_, transforming growth factor-*β*_1_; GAPDH, glyceraldehyde-3-phosphate dehydrogenase.

RETRACTED

**Table 2:** Flow cytometric analysis of normal, DMBA + croton oil, DMBA + croton oil + alcohol and DMBA + croton oil + drug-treated cells showing data of percentage of cells in different phases of cell cycle.

Series	Cell-cycle analysis by FACS			
	SubG1 (%)	G1 (%)	S (%)	G2/M (%)
Normal	32.07 ± 0.375	32.73 ± 0.565	17.44 ± 1.24	2.14 ± 0.020
DMBA + croton oil	23.39 ± 0.005	23.56 ± 0.560	25.73 ± 0.610	6.625 ± 0.375
DMBA + croton oil + alcohol	22.15 ± 0.105	28.41 ± 0.410	28.74 ± 0.640	4.76 ± 0.040
DMBA + croton oil + Sec cor 30	32.68 ± 0.310*	31.88 ± 0.995*	19.44 ± 1.16**	2.18 ± 0.28***

Values are expressed as mean ± SE. Data are the means of the results from two independent experiments. Comparisons are made between carcinogen treated and drug fed mice. *P <  .05, **P < .01; ***P < .001.
